The article "Survival Analysis of Adult Tuberculosis Disease" was retracted in 2018. Reasons: errors in the data; errors in the analysis; errors in the results or conclusions; concerns about the authorship.

# Survival Analysis of Adult Tuberculosis Disease

**DOI:** 10.1371/journal.pone.0112838

**Published:** 2014-11-19

**Authors:** Olurotimi Bankole Ajagbe, Zubair Kabair, Terry O'Connor

**Affiliations:** 1 Department of Public Health and Epidemiology, University College Cork, Cork, Ireland; 2 Mercy University Hospital, Cork, Ireland; Queen Mary Hospital, Hong Kong

## Abstract

**Background:**

We conducted a survival analysis of all the confirmed cases of Adult Tuberculosis (TB) patients treated in Cork-City, Ireland. The aim of this study was to estimate Survival time (ST), including median time of survival and to assess the association and impact of covariates (TB risk factors) to event status and ST. The outcome of the survival analysis is reported in this paper.

**Methods:**

We used a retrospective cohort study research design to review data of 647 bacteriologically confirmed TB patients from the medical record of two teaching hospitals. Mean age 49 years (Range 18–112). We collected information on potential risk factors of all confirmed cases of TB treated between 2008–2012. For the survival analysis, the outcome of interest was ‘treatment failure’ or ‘death’ (whichever came first). A univariate descriptive statistics analysis was conducted using a non- parametric procedure, Kaplan -Meier (KM) method to estimate overall survival (OS), while the Cox proportional hazard model was used for the multivariate analysis to determine possible association of predictor variables and to obtain adjusted hazard ratio. P value was set at <0.05, log likelihood ratio test at >0.10. Data were analysed using SPSS version 15.0.

**Results:**

There was no significant difference in the survival curves of male and female patients. (Log rank statistic  = 0.194, df  = 1, p = 0.66) and among different age group (Log rank statistic  = 1.337, df = 3, p = 0.72). The mean overall survival (OS) was 209 days (95%CI: 92–346) while the median was 51 days (95% CI: 35.7–66). The mean ST for women was 385 days (95%CI: 76.6–694) and for men was 69 days (95%CI: 48.8–88.5). Multivariate Cox regression showed that patient who had history of drug misuse had 2.2 times hazard than those who do not have drug misuse. Smokers and alcohol drinkers had hazard of 1.8 while patients born in country of high endemicity (BICHE) had hazard of 6.3 and HIV co-infection hazard was 1.2.

**Conclusion:**

There was no significant difference in survival curves of male and female and among age group. Women had a higher ST compared to men. But men had a higher hazard rate compared to women. Anti-TNF, immunosuppressive medication and diabetes were found to be associated with longer ST, while alcohol, smoking, RICHE, BICHE was associated with shorter ST.

The article "Survival Analysis of Adult Tuberculosis Disease" was retracted in 2018. Reasons: errors in the data; errors in the analysis; errors in the results or conclusions; concerns about the authorship.

## Introduction

Tuberculosis (TB) remains a major global health problem. It causes ill health among millions of people and ranks as the second leading cause of death from an infectious disease worldwide after human immunodeficiency virus (HIV) [1]. There were 8.6 million new TB cases in 2012 and 1.3 million TB deaths (just under 10 million among HIV negative people and 0.3 million HIV – associated TB deaths). Case-notification rates from countries with a high prevalence of tuberculosis suggest that TB may be less frequent among females. Globally, the ratio of female to male TB cases notified is 1/1·5–2·1 [2]. Females have been found to have higher TB mortality rates from birth and through the age of 29 [3]. Different explanations have been suggested to explain why women of reproductive age would have a higher progression from infection to active TB and also a higher mortality rate. An argument questioning these findings has been that women are more likely to use health services during their reproductive years, and thus are more likely to be diagnosed with TB at this time in life. [4]–[5]. Many studies have been conducted on TB; however, there are few studies that focus specifically on survival analysis of TB patients. Survival analysis is generally defined as a set of methods for analysing data where the outcome variable is the time until the occurrence of an event of interest [6]. In many medical studies, time to death is the event of interest. However, another important measure is the time between response to treatment and recurrence or relapse – free survival time (also called disease – free survival time.). The specific difficulties relating to survival analysis arise largely from the fact that only some individuals have experienced the event and, subsequently, survival times will be unknown for a subset of the study group. This phenomenon is called censoring and it may arise in the following ways: A patient has not yet experience the relevant outcome, such as relapse or death, by the time of the close of the study, or a patient is lost to follow up during the study period, or a patient experiences a different event that makes further follow – up impossible. In survival analysis, subjects are usually followed over a specified time period and the focus is on the time at which the event of interest occurs. Observations are called censored when the information about their survival time is incomplete; the most commonly encountered form is right censoring. Suppose patients were followed in a study for 20 weeks. A patient who did not experience the event of interest for the duration of the study is said to be right censored. The survival time for this person is analysis, representing a particular type of missing data, censoring that is random and non - informative considered to be at least as long as the duration of the study. Another example of right censoring is when a person drops out of the study before the end of the study observation time and did not experience the event. This person's survival time is said to be censored, since we know that the event of interest did not happen while this person was under observation. Censoring is an important issue in survival and is usually required in order to avoid bias in a survival analysis. We conducted a survival analysis of all bacteriologically confirmed cases of adult TB disease in County Cork. Ireland. The aim of this study was to estimate survival time (ST) including median time of survival and to assess the association and impact of covariates (TB risk factors) to event status and ST.

The article "Survival Analysis of Adult Tuberculosis Disease" was retracted in 2018. Reasons: errors in the data; errors in the analysis; errors in the results or conclusions; concerns about the authorship.

## Methods

This is a retrospective cohort research study which tries to analyse the survival of adult TB disease of patients that was treated in County Cork, Ireland. The study was conducted at the two main teaching hospitals that provide treatment for all TB disease in the area. Inclusion criteria were definite case of TB which was defined as a patient in whom TB had been confirmed by bacteriology (either by culture or with sputum smears positive for acid fast bacilli (AFB+). A pulmonary case which is a patient with TB disease involving the lung parenchyma. We included both smear positive pulmonary case which was defined as a patient with one or more initial sputum smear examination (direct smear microscopy) AFB+, or one sputum examination AFB+ and radiographic abnormalities consistent with active pulmonary TB as determined by a clinician. Smear negative pulmonary case, which was defined as a patient with pulmonary TB not meeting the above criteria for smear-positive disease, but with diagnosis criteria which include at least two sputum smear examinations negative for AFB; and radiographic abnormalities consistent with active pulmonary tuberculosis; and no response to a course of broad-spectrum antibiotics (except in a patient for whom there is laboratory confirmation or strong clinical evidence of HIV infection); and a decision by a clinician to treat with a full course of anti tuberculosis chemotherapy; or positive culture but negative AFB sputum examinations and Extra-pulmonary case which was defined as a patient with tuberculosis of organs other than the lungs (e.g. pleura, lymph nodes, abdomen, genitourinary tract, skin, joints and bones, meninges) with diagnosis based on one culture-positive specimen, or histological or strong clinical evidence consistent with active extra-pulmonary disease, followed by a decision by a clinician to treat with a full course of anti-tuberculosis chemotherapy. We included only patients that were 18 years and above as at the time of diagnosis and had diagnosis and treatment between January 2008 – December 2012. We excluded children under the age of 18 years and those with no specific diagnosis or confirmation of TB. Data were collected by the National Tuberculosis Notification form developed by Health Services Executive (HSE) in conjunction with the Health Protection Surveillance Centre (HPSC) in Ireland. The form is a 47-item questionnaire divided into 5- sections, namely Patient details, Socio-demographic information, Clinical details, Diagnostic details and Treatment outcome. We reviewed both the electronic medical record and the individual patient case note to collect data on gender, date of birth, age in years, current employment status, current most recent occupation, living status, country of birth, race or ethnicity, and immigration status (refugee/asylum seeker). We also collected data on Clinical details of individual patient which includes date of diagnosis, date treatment commenced, previous history of TB, Type of TB (whether pulmonary, extra-pulmonary or both), history of BCG, whether BCG scar was present or not. We collected data on the following potential risk factors, Anti-tumour necrosis factor (TNF) treatment, Immunosuppressive medication, Immunosuppressive illness, Diabetes, Born in country of high endemicity (BICHE), Residence in country of high endemicity (RICHE), Alcohol abuse, Drug misuse, Smoking, and HIV status. The treatment outcome of individual patient was also recorded i.e. completed-cured, completed – status unknown, interrupted, lost to follow up, transferred or died. Data collection started in January to December 2013. For the survival analysis, the outcome of interest was ‘treatment failure’ or ‘death’ (whichever came first). We defined treatment outcomes according to the WHO definitions of TB cases. Treatment outcomes, (expressed as a percentage of the number registered in the cohort). **Cured**: A patient who was initially smear-positive and who was smear-negative in the last month of treatment and on at least one previous occasion. **Completed treatment**: A patient who completed treatment but did not meet the criteria for cure or failure. This definition applies to pulmonary smear-positive and smear-negative patients and to patients with extra-pulmonary disease. **Died**: A patient who died from any cause during treatment. **Failed**: A patient who was initially smear-positive and who remained smear-positive at month 5 or later during treatment. **Defaulted**: A patient whose treatment was interrupted for 2 consecutive months or more. **Transferred out**: A patient who transferred to another reporting unit and for whom the treatment outcome was not known. **Successfully treated/Cured**: A patient who was cured or who completed treatment. The time to event is the time from entry into the study until the subject had a particular outcome. The date of primary diagnosis of TB was regarded as the time of entry (T0), while the date of event or death or lost to follow-up was regarded as T1, The difference between T1 and T0 was regarded as the follow up time. Subjects were said to be censored if they were lost to follow up or dropped out of the study, or if the study ended before they died or had an outcome of interest. They were counted as alive or disease-free for the time they were enrolled in the study. (Fig 1) The two-variable outcome considered was. Time variable: *Ti*  =  time at last disease-free observation or time at event. Censoring variable: *Ci*  = 1 if had the event; *Ci*  = 0 no event by time *Ti*. The primary analysis is overall survival (OS), measured from date of diagnosis of TB disease to the date of relapse or death, whichever came first. For the univariate descriptive analysis we used the nonparametric estimator of the survival function, the Kaplan Meier (KM) method that is widely used to estimate and graph survival probabilities as a function of time. The KM was used to obtain univariate descriptive statistics for survival data, including the median survival time, and compare the survival experience for the group of TB cases by gender and age groups. Survival Function S (t): Defined as the probability of surviving at least to time t. (Graph of S (t) against t) (Fig 2). Hazard Function h (t): Defined as the conditional probability of experiencing an event at time t having survived to that time. (Fig 3). For multivariable analyses, Cox regression models with forward and backward stepwise selection (inclusion criteria: p value of the score test <0.05, exclusion criterion p-value of the likelihood ratio test >0.10 were used to analyse the association or effect of following potential predictor variables. Gender (Categorical, coded 1: Male, 0: Female), Marital status (categorical & coded 1: Single, 2: Married, 3: Widowed, 4: Divorced 5: Unknown, 6: Others.). Age (Continuous & coded 1: 18–30, 2: 30–45, 3: 45–59, 4: 59–79, 5: 80 and above. Sex (Categorical & coded 1: Male, 0: Female), Marital status (Categorical & coded 1: Single, 2: Married, 3: Widowed, 4: Others, 5: Unknown, 6: Divorced,), Ethnicity/Race (Categorical & coded 1: Black, 2: White Black, 3: South Asian descent, 4: East/South Asian descent, 5: Others. Occupation (Categorical & coded 1: Unemployed, 2: Healthcare, 3: Environmental Design, 4: Engineering, 5: Administration/Business, 5: Education, 6: Others). Employment status (Categorical & coded: 1: Paid employment, 2: Housewife/husband, 3: Unemployed, 4: Retired, 5: Student, 6: Others, 7: Unknown.). Living status (Categorical & coded 1: Home (Private/Rented), 2: Homeless, 3: Hostel, 4: Prison), Country of birth (Categorical & coded 1: Ireland, 2: Others.), Refugee/Asylum seeker. (Categorical & coded 1: Yes, 2: No, 0: Unknown)

**Figure 1:** Censored cases.

The article "Survival Analysis of Adult Tuberculosis Disease" was retracted in 2018. Reasons: errors in the data; errors in the analysis; errors in the results or conclusions; concerns about the authorship.

**Figure 2:** Plot of the Kaplan Meier Survival function curve for the data.

**Figure 3:** Plot of the Cumulative Hazard function for the data to test the assumption of Cox Proportional Hazard.

Analysis was performed using SPSS software, version15.0. The overall differences between estimated survival curves of patients by gender (males versus females), and different age group were calculated by the log-rank test. We were unable to get a written informed consent from participant in this study so the patient record was anonym zed prior to analysis.

## Results

A total of 647 patients were included in this study. Male patients were 413 (66.2%), while female patients accounts for 234 (33.8%). The mean age was 49 years (Range: 18–112). The patients marital status showed that a total of 277 (40%) patients were single, 265(38%) were married, 39 (5%) were widowed and 5 (1%) were divorced. The result of country of birth showed that 314 (45%) were Irish, while 379 (44.3%) were foreign born. Employment status of patients showed that 131 (18.9%) were on paid employment, 128 (18.5%) were unemployed, 59 (8.5%) were retired while 5 (1%) were students. Patients living status showed that half 347 (50%) were living in private/rented home. The result of patients ethnicity showed that close to half 335 (48.3%) of the patients were white, while 48 (7%) were black. 262 (38%) had diagnosis of PTB, 27 (4%) were EPTB while 17 (3%) had both PTB and EPTB. The results are as presented in Table 1.

**Table 1:** Study Participants Characteristics.

Characteristics	Number of Patients	% of Patients
**Age in Years**		
Mean	49	
Range	18–112	
**Gender**		
Female	234	33.8
Male	413	66.2
**Marital Status**		
Single	277	40
Married	265	38.2
Widowed	39	5.6
Divorced	5	0.7
Unknown	51	15.5
**Occupation**		
Unemployed	11	1.6
Healthcare	22	3.6
Environmental design	3	0.4
Engineering	13	1.9
Administration/Business	17	2.5
Education	22	3.2
Others	180	26
Unknown	425	425
**Country of birth**		
Ireland	314	45.3
Others	379	4.7
**Employment Status**		
Paid employment	131	18.9
Housewife/husband	15	2.2
Unemployed	28	18.5
Retired	59	8.5
Student	5	0.7
Others	13	1.9
Unknown	342	49.4
**Living Status**		
Home (Private/rented)	347	50.1
Homeless	4	0.6
Hostel	1	0.1
Prison	1	0.1
Unknown	376	48.1
**Ethnicity**		
Black	48	6.9
White	335	48.3
South Asian descent	2	0.3
East/South Asian descent	4	0.6
Others	3	0.4
Unknown	301	43.4
**Refugee/Asylum seeker**		
Yes	16	2.3
No	301	43.4
Unknown	376	54.3
**Diagnosis**		
Pulmonary (PTB)	262	37.8
Extra-pulmonary (EPTB)	27	3.9
Both. (PTB + EPTB)	17	2.5
**Study Hospital**		
CUH	152	21.9
MUH	495	71.4

The result of the univariate descriptive statistics for the survival data are as shown in Table 2. It shows that out of a total number of 647 patient only 62 had an event. Out of those who had an event, 41 were men while 21 patients were women. Also, out of 413 men only 41 had an event and 372 (90%) were censored. Whereas out of the 234 women only 21 had an event and 213 (91%) were censored. The OS time was 209 days (95% CI: 72–346).

The article "Survival Analysis of Adult Tuberculosis Disease" was retracted in 2018. Reasons: errors in the data; errors in the analysis; errors in the results or conclusions; concerns about the authorship.

**Table 2:** Descriptive Statistics of Survival Data (SPSS Output of Kaplan-Meier Estimator).

Covariates	Mean Survival Time(days)	95% CI	Median Survival time	95% CI	Log rank	Df	Sig
**Gender**							
Female	385	77–694	49	16.5–81.5			
Male	69	49–89	52	31.7–72.3	0.194	1	0.66
**Alcohol**							
Yes	101	53–149	77	26–127			
No	509	142–876	96	28–144	1.8	1	0.18
**Smoking**							
Yes	102	62–144	68	31.5–104			
No	601	58–1144	59	0.0–723	0.1	1	0.75
**Anti-TNF**							
Yes	128	54–202	68	50–86			
No	51	29–72	41	17–65	1.4	1	0.23
**RICHE**							
Yes	44	25–64	25	0.0–57.3			
No	369	108–630	77	35.8–118.3	0.5	1	0.5
**BICHE**							
Yes	52.5	33.4–71	59	6.4–111			
No	370	109–631	77	35.8–118	0.2	1	0.7
**IMMSD**							
Yes	554.9	116–993	68	0.0–740			
No	107	64–149.7	96	29–162	0.5	1	0.5
**Diabetes**							
Yes	156	79–232					
No	81.7	48.5–114	59	17.8–100	0.4	1	0.6

*Since the significance value was greater than 0.05, we concluded that the association between covariates and survival time was not statistically significant

*(No statistics were computed for the following covariate because all cases were censored.

(Employment status, living status, marital status, occupation, ethnicity, refugee, TB type, TB hx, BCG, SCAR, IMMSI and HIV status).

We compare the survival function of the subjects according to gender by plotting the Kaplan –Meier (KM) graph. The KM graph displays the cumulative survival function on a linear scale by gender (Fig 2). The survival curve of men were lower than that of women, which means that men have a higher probability of surviving (not experiencing an event) than women. The overall median survival time was 51 days (35.7–62.3). However, in the graph of Fig 3 which displays the cumulative hazard curves of men and women. The graph showed that women had a lower cumulative hazard curve compared to men, which means that women had a higher probability of experiencing an event which in this case is either treatment failure or death compared to men. Table 2 shows the result of descriptive statistics of covariates with ST. The result showed that women had a longer ST compared to men, the mean ST for women was 385 days while that of men was 69 days. Also, patients with Anti-TNF had ST of 128 days while those with no Anti-TNF was 51 days, patients with immunosuppressive drug (IMMSD) had ST of 554 days, while those with no immunosuppressive drug was 107 days, also those patient with diabetes had ST of 156 days compared to 82 days if patient was not diabetic. These findings showed that these covariates were associated with longer ST. The result also showed that the p-value of the association was 0.66 and since this was greater than 0.05, so we concluded that the association was not statistically significant. The association of all other covariates with ST and significance level were as shown in the table.

The article "Survival Analysis of Adult Tuberculosis Disease" was retracted in 2018. Reasons: errors in the data; errors in the analysis; errors in the results or conclusions; concerns about the authorship.

We also compared the survival function by level of factor. The comparisons of survival curve for the different age category was performed using Log rank test. This was used to test the hypotheses that there was no difference between the population survival curves according to age category. (i.e the probability of an event occurring at any point is the same for each population). The result of the comparison are as shown in Table 3. It shows that the overall comparison was 0.7 and since the significance value for the comparison was more than 0.05, we also concluded that the survival curves are the-same across age group. The graph of the KM plot for different age category is as shown in Fig 4. The graph shows that age group 18–30 had the lowest survival curves while 30–45 age category had the highest curve. The hypothesis was accepted because the score showed no significant difference as p value was more than 0.05 for age category.

**Figure 4:** Plot of KM for Age Category.

**Table 3:** Comparison for control Variable: Age.

Comparison	Wilcox on (Gehan)Statistic	df	Sig
Overall comparison Pairwise comparison (Age 1)	1.337	1	0.720
2	0.000	1	0.991
3	0.870	1	0.351
4	0.75	1	0.78
Age 2			
1	0.000	1	0.991
3	0.817	1	0.336
4	0.678	1	0.410
Age 3			
1	0.870	1	0.351
2	0.817	1	0.366
4	0.165	1	0.684
Age 4			
1	0.75	1	0.784
2	0.678	1	0.410
3	0.165	1	0.684

Comparison is exact.

*Age 1: 18–30, Age 2: 30–45, Age 3: 45–60, Age 4: Over 60.

(This is the table than compares level of factor. Since the significance value for the overall comparison was more than 0.05, we concluded that the survival curves are the-same across age group).

The article "Survival Analysis of Adult Tuberculosis Disease" was retracted in 2018. Reasons: errors in the data; errors in the analysis; errors in the results or conclusions; concerns about the authorship.

The model that describes the potential association between covariates and survival time was analysed using a Cox proportional hazard model. This enables us to determine the difference between the survival times of the different group to be tested with other potential explanatory variables. In this model, the dependent variable was the ‘hazard’. The hazard is the probability of experiencing an event which in this case was ‘treatment failure or death’ given that the patient had survived up to a given point in time or the risk of death at that moment. The result of the association is as shown in Table 4. Looking at the table, the value Exponential (B) for person born in countries of high endemicity (BICHE) means that the TB hazard for that patient was 6.3 times that of a patient that was not BICHE. Other covariates that were associated with TB hazard were Drug misuse (2.2 times), Smoking (1.8 times), Alcohol (1.8 times) and Immunosuppressive medication (3.0 times). In Cox model, no assumption is made about the probability distribution of the hazard, however, it is assumed that the proportional hazard is constant over time. This assumption t was inspected by looking at a graph showing the logarithm of the estimated cumulative hazard function. The assumption is equivalent to assuming that the difference between the logarithms of the hazards for both gender did not change with time, or equally that the difference between the logarithms of the cumulative hazard functions was constant. Figure 3 is the graph for the data. The lines for male and female patient were roughly parallel, suggesting that the proportional hazards assumption is reasonable in this case.

**Table 4:** SPSS Output for Covariates with Survival Time.

	B	SE	Wald	df	Sig	Exp B	Lower	Upper
Gender	.105	.623	.028	1	.867	1.110	.327	3.766
Age	−.029	.018	2.514	1	.113	.971	.937	1.007
Marital	5.468	88.146	.004	1	.951	236.978	.000	2.53977
Anti-TNF	−.445	1.034	.185	1	.667	.641		
IMMSD	1.097	2.185	.252	1	.616	2.996		
IMMSIL	−1.436	2.182	.433	1	.510	.238		
BICHE	1.836	1.193	2.370	1	.124	6.271	.606	64.932
RICHE			.	0^a^	.			
Diabetes	.191	.729	.069	1	.793	1.210	.290	5.052
Smoking	.606	.936	.419	1	.518	1.833	.293	11.482
Alcohol	.589	.740	.634	1	.426	1.803	.423	7.691
Drug Misuse	.774	.601	1.657	1	.198	2.168	.667	7.043
TB hx	−.186	.946	.038	1	.844	.831	.130	5.303
BCG	−1.074	1.280	.704	1	.401	.342	.028	4.197
BCG SCAR	1.035	1.191	.756	1	.385	2.816	.273	29.083
HIV	0.18	0.261	0.477	1	0.49	1.197	.718	1.996
Refugee	−.533	1.559	.117	1	.733	.587	.028	12.466
Ethnicity	−.408	.978	.175	1	.676	.665	.098	4.516
Living Status	−4.313	406.196	.000	1	.992	.013	.000	.
Occupation	−.221	.212	1.085	1	.298	.802	.529	1.215
Employment Status	−.443	.394	1.262	1	.261	.642	.297	1.391

**95% CI for Exp (B).**

The article "Survival Analysis of Adult Tuberculosis Disease" was retracted in 2018. Reasons: errors in the data; errors in the analysis; errors in the results or conclusions; concerns about the authorship.

*Test of Model Coefficients: −2 Log likelihood: 119, Chi-square:16.172, df: 20, p-value: 0.706.

(The overall p value was more than 0.05, so we concluded that no covariate has a significant impact on survival time.).

## Discussion

The first objective of this study was to examine the distribution of the follow up time to event among the population. The result of the Life table and KM curve showed that the distribution of follow up time to event by age category and gender follows a normal distribution.

The second objective was to estimate survival function including the median survival time and compare the survival curves by groups. The KM survival curves in this data showed a steep decline in the early days of receiving treatment, this indicates poor prognosis from the disease. Also, we found out that the number of men who had TB were far more than women, men accounted for about three quarter of the total population, whereas only one quarter were women, which means that TB is common among men. The probable reason might be due to men's general lifestyle. Majority of men likes to smoke cigarettes, drink alcohol etc and these are one of the major risk factors for TB [7]. W.H.O publication on TB and gender documented that more men than women were diagnosed with TB and died from it. [1], [12], [13], [14]. TB is nevertheless a leading infectious cause of death among women [8]–[10]. Annually, about 700 000 women died of TB, and over three million contract the disease, accounting for about 17 million Disability Adjusted Life Years (DALY) [11], [15]. The result also showed that the estimated OS was 209days while the median was 51 days this findings is similar with some other studies. In a study conducted by Oursler et al 2002 showed that the median time to event was 39 days in TB patient and survival time was 202 days [16]. TB among mothers has been found to be associated with a six-fold increase in perinatal deaths and a two-fold risk of premature birth and low birth-weight for age [14]. We compared the survival curves by gender and by age category. We found out that there was no significant difference in the survival curves of male and female patients. and among different age group. However, age has been identified as an important risk factor for death in TB patients. Different studies showed that age was a factor that is affecting survival of TB patients. According to Hoorne et al in Washington state, mortality was independently associated with increasing age [17]. A study in Maryland community-based cohort of patients with drug susceptible pulmonary TB also showed that age was strongly associated with risk of death. This study showed that age 18–30 had the highest treatment failure and mortality. One of the most important causes of unsuccessful treatment is irregularity and loss to follow-up which may be due to patients being transferred to another unit. Generally, treatment failure may also be due to poor compliance to medication by the patients. A report from the USA showed that non compliance was associated with a 10 – fold increase in the occurrence of poor treatment outcomes and accounted for most treatment failures. This study also aimed to determine the potential risk factors associated with length of survival. We used the Cox's proportional hazards model as the analogous to multiple regression models that enables the difference between survival times of particular groups of patients to be tested while allowing for other factors. In this model, the response (dependent) variable is the ‘hazard’. We found that Anti TNF, IMMSD and diabetes were associated with longer survival time while Smoking, Alcohol, RICHE and BICHE were associated with longer survival time. Several systematic reviews have found substantial evidence that these risk factors were associated with an increased risk of TB infection and TB disease [18]. There was also some evidence (albeit less robust), regarding the adverse effects of active smoking on TB mortality and on TB outcomes in patients in whom, the disease is established. Active smoking had been found to be associated with lower treatment adherence, slower smear conversion, TB treatment failure, relapse and death during or after treatment [19]–[20]. Furthermore, the joint effects of smoking, TB and HIV greatly increase the risk of chronic obstructive pulmonary disease in the long term [11]. The introduction of smoking cessation services into TB programs has therefore been advocated by several international bodies [12].

The article "Survival Analysis of Adult Tuberculosis Disease" was retracted in 2018. Reasons: errors in the data; errors in the analysis; errors in the results or conclusions; concerns about the authorship.

## Conclusion

There was no significant difference in survival curves of male and female and among age group. Women had a longer ST compared to men.

But men had a higher hazard rate compared to women. Anti-TNF, IMMSD and diabetes were found to be associated with longer ST, while alcohol, smoking, RICHE, and BICHE were associated with shorter ST. The association was however not statistically significant as the p-value was greater than 0.05.

## Limitations

This study has a number of limitations, firstly, generally in survival analysis; there is assumption of homogeneity of treatment and other factors during the follow – up period, however in this study the case mix changes over the period of recruitment. The KM method assumes that the survival probabilities are the same for subjects recruited early and late in the study. On average, subjects with longer survival times would have been diagnosed before those with shorter times and changes in treatment, earlier diagnosis and some other changes over time may lead to spurious result. Also, children under the age of 18 years were excluded from the study because they did not meet the inclusion criteria as a result we are unable to apply the result of this study to children with TB. Another limitation is the fact that some of the patient's medical record did not have all the required information needed for this study; hence we are limited by only the information at our disposal. For example treatment outcomes of patients were not recorded in some of the notes, so it was very difficult to know the status of that patient after treatment. We also noted some inconsistency in the information. that are contradictory on the patient's medical record making it somehow difficult to know the correct status of a patient at particular time, a good example of this is that they may record that a patient is non-smoker in one place and in another place it may be recorded that the patients is a smoker.

### Ethic Approval

Approval to undertake this study was sought and granted by the ‘Clinical Research Ethic Committee of the Cork Teaching Hospital' (CREC). We were unable to get a written inform consent from participant in this study so the patient record was anonymized prior to analysis.

#### Implication to policy and clinical practice

This study recommended that hospitals maintain a standardised method of assessment of TB patient by using appropriate assessment procedures. We advise that they start using the enhanced TB notification form that was used in this study during patient's assessment process. This will not only improve the quality of care to the patient, but will also facilitate accurate diagnosis and effective documentation that will be useful for other researchers in the area of TB in future.
